# College Smart Classroom Attendance Management System Based on Internet of Things

**DOI:** 10.1155/2022/4953721

**Published:** 2022-07-05

**Authors:** Mingtao Zhao, Gang Zhao, Meihong Qu

**Affiliations:** Architectural Engineering School, Qingdao Huanghai University, Qingdao, Shandong 266427, China

## Abstract

Since entering the information age, educational informatization reform has become the inevitable trend of the development of colleges and universities. The traditional education management methods, especially the classroom attendance methods, not only need to rely on a large number of manpower for data collection and analysis but also cannot dynamically monitor students' attendance and low efficiency. The development of Internet of things technology provides technical support for the informatization reform of education management in colleges and universities and makes the classroom attendance management in colleges and universities have a new development direction. In this study, a college smart classroom attendance management system based on RFID technology and face recognition technology is constructed under the architecture of the Internet of things, and the corresponding simulation experiments are carried out. The experimental results show that the smart classroom attendance management system based on RFID technology can accurately identify the absence and substitution of students and has the advantages of fast response and low cost. However, its recognition is easily affected by obstructions, which requires students to place identification cards uniformly. The smart classroom attendance management system based on face recognition technology can accurately record and identify the situation of students entering and leaving the classroom and identify the situations of being late and leaving early, absenteeism, and substitute classes. The experimental results are basically consistent with the sample results, and the error rate is low. However, the system is easily affected by environmental light, students' sitting posture, expression, and other factors, so it cannot be recognized. Generally speaking, both can meet the needs of classroom attendance in colleges and universities and have high accuracy and efficiency.

## 1. Introduction

The development of information technology and Internet of things technology has promoted the pace of educational informatization reform. The informatization development of educational management has also become one of the focuses of attention and research in colleges and universities. The development of college education management methods and mechanisms needs to measure the effectiveness and rationality of daily teaching through real and scientific data, in which student classroom attendance is an important part of college education management [1]. Classroom attendance includes student attendance and teacher attendance. It can not only reflect students' learning behavior but also reflect the authenticity and effectiveness of teachers' teaching classroom and provide important basic data information for teaching reform. The collection of classroom attendance data is closely related to the classroom attendance technology and methods. The traditional classroom attendance method is mainly manual attendance. Such attendance methods not only can dynamically grasp the attendance status of students, but also is prone to errors and omissions. It also needs to repeatedly test the attendance information, which consumes a lot of manpower and materials [2]. At the same time, manual attendance records are generally recorded, sorted, and kept by teachers, so it is not easy for students to understand their attendance. Therefore, the traditional classroom attendance method can meet neither the needs of students and teachers nor the requirements of the development of information technology in colleges and universities [3].

The development of Internet of things technology provides a new development direction for colleges and universities to build information-based classroom attendance system and mechanism. Many colleges and universities are also constantly trying new technologies in the process of building smart classrooms. Therefore, this study proposes the research on a college smart classroom attendance management system based on the Internet of things, constructs the classroom attendance management system based on RFID technology and face recognition technology, and carries out the corresponding simulation test. This study is mainly divided into three parts: the first part expounds on the development of classroom attendance technology in colleges and universities; the second part is to build a classroom attendance management system based on RFID technology and face recognition technology under the framework of the Internet of things; the third part is the test and result analysis of classroom attendance management system based on RFID technology and face recognition technology.

Under the architecture of Internet of things, this study constructs an attendance management system of intelligent classroom in colleges and universities based on RFID technology and face recognition technology and carries out the corresponding simulation experiments. Research and innovation contributions are as follows: (1) The intelligent classroom attendance management system based on RFID technology can accurately identify the absence and substitution of students. It has the advantages of fast response and low cost. (2) The intelligent classroom attendance management system based on face recognition technology can accurately record and identify the situation of students entering and leaving the classroom and identify the situation of being late and leaving early, absenteeism, and substitute classes. The experimental results are basically consistent with the sample results, and the error rate is low. The research provides technical support for the development of Internet of things technology and the reform of educational management informatization in colleges and universities and makes the classroom attendance management in colleges and universities have a new development direction.

## 2. Development of Classroom Attendance Technology in Colleges and Universities

The development of college attendance technology is closely related to the development of information technology and Internet technology. Before the wide application of information technology and Internet technology, classroom attendance was mainly based on traditional manual attendance; that is, the arrival of paper signs was used to record the attendance of students and teachers in class, and then the relevant personnel carried out data statistics and analysis after class [4]. Teachers will also conduct random roll calls and multiple roll calls in class according to the actual situation to monitor students' classroom attendance. To a certain extent, this attendance method restricts the occurrence of students' behaviors such as being late, leaving early, and absenteeism and improves the management of students. In addition, the teaching method of colleges and universities is different from that of middle schools. There is no fixed class. Manual attendance can help teachers know and understand students, shorten the distance between students and teachers, and improve the communication between teachers and students [5]. However, with the expansion of the scale of colleges and universities and the increase of the number of students, the way of manual attendance will take up a lot of time, and the accuracy and efficiency of attendance will be reduced. At the same time, the way of manual attendance cannot realize the timely feedback and dynamic tracking of relevant data, and the head teacher cannot timely understand and master the situation of students' classroom attendance [6].

With the development and application of computer technology, classroom attendance also began to enter the information age. Electronic communication technology and computer technology provide technical support for the informatization of classroom attendance. Some scholars propose to combine campus magnetic card or IC card with computer technology to collect and store campus card and student information through the attendance equipment that can be read, so as to be applied to the attendance system [7]. Other scholars have combined RFID technology to design a system that can carry out attendance and recording simply, quickly, and automatically, which improves the accuracy, efficiency, and timeliness of attendance technology [8]. As campus cards and other cards are forged, fraudulently used, and embezzled, which reduces the accuracy and authenticity of attendance data, someone developed biometric attendance technology based on computer technology and biological science and technology [9]. Biometric attendance technology is composed of computer technology, optics, acoustics, biosensors, statistical principles, and other discipline technologies. It mainly verifies personal identity through the inherent behavior and physiological characteristics of human body. The common ones are fingerprint recognition, iris recognition, and so on [10, 11].

With the development of mobile Internet technology and equipment, the smart campus and smart classroom have become important development models of colleges and universities and put forward higher requirements for attendance technology and methods of colleges and universities [12]. On the basis of big data, Internet of things, and other information technologies, college classroom attendance combines intelligent mobile devices to build a new generation of classroom attendance system [13]. Some scholars have built an intelligent classroom attendance system with Internet of things technology as the core and verified its good system stability through experiments [14]. On the basis of mobile Internet, other scholars have realized the active and random data collection of classroom attendance information by using intelligent mobile terminal equipment, bluetooth, QR code, app, etc., which can feed back and track the information data in real time [15]. However, such attendance methods must be used in an environment that can connect to the network, and it is also unable to identify the substitute class. Therefore, some scholars proposed to integrate radio frequency identification technology into the classroom attendance system and constructed RFID-based automatic identification campus attendance technology, which can carry out real-time senseless data collection [16]. Other scholars have built a classroom attendance system based on face recognition technology, which improves the uniqueness and exclusivity of attendance and reduces the number of clock outs while ensuring the accuracy of classroom attendance [17]. However, face recognition technology needs to build a corresponding database. As in the early stage of the development of this technology, the technology has certain limitations, high management cost, and easy to be affected by environmental factors [18]. With the deepening of education informatization reform in colleges and universities, colleges and universities are constantly innovating and practicing the classroom attendance system according to their own actual situation and needs and are also constantly adjusting and improving the education management mechanism, so as to provide more convenient, fast, and reliable information services for teachers and students [19].

## 3. College Smart Classroom Attendance Management System Based on Internet of Things

The classroom attendance management system is based on Internet of things technology. The Zige system is convenient for teachers to collect and manage students' attendance information and improve the accuracy of Zige's 3G sensor network, which not only saves students' time and attendance but also improves students' attendance and management. With the continuous development of Internet, Internet of things, and information technology, colleges and universities have been exploring and studying efficient and convenient smart classroom attendance methods that can analyze classroom attendance data in the practice of building smart classroom, so as to provide multidimensional and diversified decision support for the development of smart classroom in colleges and universities [20]. At the same time, we also need to take into account the actual needs of smart classroom in colleges and universities, the software and hardware conditions required by attendance methods, technical feasibility, and economic feasibility. Therefore, the classroom attendance management system based on RFID technology and the classroom attendance management system based on face recognition technology have become the choice of many colleges and universities. As the core content of face recognition, feature extraction and comparison recognition are to use computer technology to locate the location of biological key points. After geometric and optical corrections, the feature key points that can be compared are extracted and compared with the facial texture code of the face database. Finally, the automatic processing technology of individual identification is carried out.

### 3.1. Construction of College Classroom Attendance Management System Based on RFID Technology

The traditional classroom attendance card swiping method in colleges and universities can neither control the number of students in the classroom and the situation of students being late and leaving early in real time nor identify problems such as one person with multiple cards. The classroom attendance management system based on RFID technology can realize the way of real-time and efficient roll call and information attendance and master the attendance of the classroom in real time. As shown in Figure 1, it is the overall block diagram of the classroom attendance management system based on RFID technology.

RFID technology can realize indoor real-time positioning in a large range of coverage without contact and has the advantages of high visibility, convenience, and low cost. For indoor positioning based on RFID technology, the basic coordinates need to be selected according to the specific situation of the classroom, and the corresponding calculation is carried out through the coordinates. Considering that there will be a multipath effect in positioning through the distance between the electronic tag and the receiver, which will affect the accuracy of positioning coordinates, this study uses the strength of the relative received signal for indoor positioning, and its calculation is shown in the following formula:

(1) $$\begin{array}{c} PL\left(d\right)=pl\left(d_{0}\right)-10n\mathrm{lg}\left(\frac{d}{d_{0}}\right)-X_{0}. \end{array}$$

In the formula, the distance between the electronic tag and the reader is expressed as *d*, the reference distance is expressed as *d*_0_, the environmental parameter is expressed as *n*, the signal strength at the distance *d* between the electronic tag and the reader is expressed as *PL*(*d*), and the signal strength at the reference distance is expressed as *pl*(*d*_0_).

The coordinate position of the label to be tested is set as (*x*, *y*) and the position of the reader-writer as (*X*_*i*_, *Y*_*i*_). When the position is known, the distance between the label to be tested and the *i* reader-writer is shown in the following formula:

(2) $$\begin{array}{c} d_{i}=\sqrt{{\left(x_{i}-x\right)}^{2}+{\left(y_{i}-y\right)}^{2}}. \end{array}$$

If there is an intersection *A* in the effective area of two readers and writers, and there is also an intersection outside the area, then the *A* point is reasonable. The average value of all solutions is calculated to obtain the final solution of each label, as shown in the following formulas:

(3) $$\begin{array}{c} X=\sum_{i=1}^{I}\frac{X_{i}}{I}, \end{array}$$

(4) $$\begin{array}{c} Y=\sum_{i=1}^{I}\frac{Y_{i}}{I}. \end{array}$$

The label value obtained according to the formula is (*X*, *Y*), which is converted into the reference coordinates of the setting area to obtain the specific position of the label seat.

Friis path loss model realizes positioning through Frith transmission formula in a free propagation model, as shown in the following formula:

(5) $$\begin{array}{c} P_{r}=P_{t}\cdot G_{r}\cdot G_{t}\cdot L_{\text{path}}. \end{array}$$

The model power received by the passive tag is expressed as *P*_*r*_, the transmission power of the reader is expressed as *P*_*t*_, the radiation radius of its corresponding reading and writing area is expressed as *R*, the antenna gain of the reader is expressed as *G*_*r*_, the antenna gain of the tag is expressed as *G*_*t*_, and the path loss is expressed as *L*_path_. The expression is shown as follows:

(6) $$\begin{array}{c} L_{\text{path}}={\left(\frac{\lambda }{4\pi R}\right)}^{2}. \end{array}$$

Combining formulas (5) and (6)

(7) $$\begin{array}{c} P_{r}=P_{t}\cdot G_{r}\cdot G_{t}\cdot {\left(\frac{\lambda }{4\pi R}\right)}^{2}. \end{array}$$

The logarithm of formula (7) is obtained as follows:

(8) $$\begin{array}{c} P_{r}=P_{t}+G_{r}+G_{t}+20\mathrm{lg}\left(\frac{\lambda }{4\pi R}\right). \end{array}$$

Due to the amplitude fading caused by human interference or obstruction in the indoor environment, the reception power of passive tags is reduced, resulting in the problem of missing reading. Therefore, formula (8) is modified as follows:

(9) $$\begin{array}{c} P_{r}{}^{\prime }=P_{t}+G_{r}+G_{t}-20\mathrm{lg}\left(\frac{4\pi R}{\lambda }\right)-\left|X_{\sigma }\right|. \end{array}$$

The Gaussian white noise is expressed as *X*_*σ*_, its standard deviation is expressed as *σ*, and the actual received power of the tag is expressed as *P*_*r*_′.

Each seat in the classroom represents the corresponding target area. In principle, each target area corresponds to only one electronic label. When multiple electronic labels appear on the same seat, students may brush on behalf of others. As shown in Figure 2, it is the effect diagram of antiproxy brushing of college classroom attendance management system based on RFID technology.

The traditional attendance management is time consuming, laborious, and inefficient, and the information is not timely, which cannot meet the management requirements of modern colleges and universities. Therefore, it is necessary to adopt the student attendance management system based on the campus network to automatically collect student attendance information through RFID (radio frequency identification) technology. To avoid that teachers' roll call takes up classroom teaching time and improve teaching efficiency, the convenience of students' leave and the efficiency of management approval is improved through online leave and approval. Students, teachers, and teaching management departments share attendance information through the campus network to increase the transparency of information and improve the management quality of management departments. The attendance management system will automatically calculate the number and position of electronic tags according to the RFID antenna in the classroom, so as to obtain the precise position of each electronic tag in the classroom and identify normal seats, empty seats, and proxy brushing seats with multiple cards. However, if students put the card in their schoolbag or pocket, it may affect the accuracy of measurement. In actual use, students will be required to place the card in a certain position on the desktop to reduce missing reading.

### 3.2. Construction of College Classroom Attendance Management System Based on Face Recognition Technology

With the development of Internet of things technology, face recognition technology is widely used in the smart campus of colleges and universities. Face recognition technology combined with wireless network technology can realize classroom attendance check-in, detect students' late and early leave, absenteeism, substitute class, etc., and effectively and accurately record students' access to the classroom. The face recognition technology in this study is based on the Harr feature to detect the face; that is, the integral graph method is used to calculate many matrix features contained in the detection window. Let the sum of the luminance values of the rectangular area composed of the image starting point and point *i*(*x*, *y*) be expressed as *s*(*x*, *y*), and it will be saved in the memory as an integral value. When the vertical and horizontal coordinates of the image to be calculated exceed the sum of the lighting degrees of all pixels of point *i*(*x*, *y*), it can be calculated as long as it traverses all points of the original image once, as shown in the following formula:

(10) $$\begin{array}{c} s\left(x,y\right)=s\left(x-1,y\right)+s\left(x,y-1\right)-s\left(x-1,y-1\right)+i\left(x,y\right). \end{array}$$

In order to reduce the interference and recognition influence on the classroom attendance system and improve the recognition efficiency and accuracy, it is necessary to preprocess the image. By calculating the weighted average of the red specific gravity, green specific gravity, and blue specific gravity of the color image, the transformation of the image gray scale is completed. The calculation formula is shown as follows:

(11) $$\begin{array}{c} \text{gray}=0.299*R+0.587*G+0.144*B. \end{array}$$

Then, the image is histogram equalized and its new pixel value is calculated, as shown in the following formula:

(12) $$\begin{array}{c} s_{k}=\sum_{j=0}^{k}\frac{n_{j}}{n}, \end{array}$$

where *k*=0,1,2,…, *L* − 1, the total number of image pixels is expressed as *n*, the number of pixels of the current gray level is expressed as *n*_*j*_, and the total number of possible gray levels of the image is expressed as *L*.

Because the gray scale of LBP operator has good robustness and is not affected by lighting conditions, it has a fast computing speed and can analyze images in a complex real-time environment. Therefore, the university classroom attendance management system based on face recognition technology in this study is based on the LBP method for image feature extraction. LBP is initially set in the 3 × 3 pixel field, and the gray values of nine pixels in the field are extracted. The central pixel is selected as the threshold and the gray value is compared with the other eight adjacent pixels. When the central pixel is lower than the gray value of the adjacent pixel, the adjacent pixel is recorded as 1; otherwise, it is 0. The calculation formula of LBP value of the central pixel of the neighborhood is shown as follows:

(13) $$\begin{array}{c} LBP\left(x_{c},y_{c}\right)=\sum_{p=0}^{p-1}2^{p}s\left(i_{p}-i_{c}\right). \end{array}$$

In the formula, the central pixel of the neighborhood is expressed as (*x*_*c*_, *y*_*c*_), its pixel value is expressed as *i*_*c*_, other pixel values in the field are expressed as *i*_*p*_, and the symbolic function is expressed as *s*.

In order to enable LBP to better extract texture features from large-scale images, the LBP operator is improved to a circular LBP operator; that is, it is assumed that it contains eight sampling points in the 5 × 5 neighborhood, and the coordinate value calculation formulas of each sampling point are shown as follows:

(14) $$\begin{array}{c} x_{p}=x_{c}+R\text{cos}\left(\frac{2\pi p}{p}\right), \end{array}$$

(15) $$\begin{array}{c} y_{p}=y_{c}+R\text{sin}\left(\frac{2\pi p}{p}\right), \end{array}$$

where the center point of the neighborhood is expressed as (*x*_*c*_, *y*_*c*_) and a sampling point is expressed as (*x*_*p*_, *y*_*p*_).

When the university smart classroom attendance management system performs face recognition through LBPH algorithm, it needs to initialize parameters first and then LBP coding; that is, (*x*, *y*)_*n*_ is set as the corresponding pixel offset coordinate in the *n* field, and its calculation formula is shown as follows:

(16) $$\begin{array}{c} \left\{\begin{array}{c} x_{n}=-\text{radius}\times \text{sin}\left(2.0\times \pi \times \frac{n}{\text{neighbors}}\right),\\ y_{n}=-\text{radius}\times \text{cos}\left(2.0\times \pi \times \frac{n}{\text{neighbors}}\right). \end{array}\right. \end{array}$$

The *n* field gray value of all pixel coordinates is calculated through bilinear difference, and the coded value is calculated according to the following formula:

(17) $$\begin{array}{c} lbp{\left(x,y\right)}_{n}=\left\{\begin{array}{c} 1\ldots \left(\text{gray}{\left(x,y\right)}_{n}\leq \text{gray}\left(x,y\right)\right),\\ 0\ldots \left(\text{gray}{\left(x,y\right)}_{n}>\text{gray}\left(x,y\right)\right). \end{array}\right. \end{array}$$

The calculation formula of LBP coding value of all pixels contained in each submodule is shown as follows:

(18) $$\begin{array}{c} lbp\left(x,y\right)=\sum_{n=0}^{\text{neighbors}-1}lbp{\left(x,y\right)}_{n}\times 2^{n}. \end{array}$$

The histogram is calculated. The calculation formula of the width and height of each grid in the image is shown as follows:

(19) $$\begin{array}{c} \left\{\begin{array}{c} w\_\text{grad}=LBP_{i}\cdot \text{cols}/\text{gridx},\\ h\_\text{grad}=LBP_{i}\cdot \text{rows}/\text{gridx}. \end{array}\right. \end{array}$$

The similarity between two histograms is calculated by the card method, as shown in the following formula:

(20) $$\begin{array}{c} d\left(H_{1},H_{2}\right)=\frac{{\left(H_{1}-H_{2}\right)}^{2}}{H_{1}+H_{2}}. \end{array}$$

## 4. Test and Results of College Smart Classroom Attendance Management System Based on Internet of Things

### 4.1. Test and Results of College Classroom Attendance Management System Based on RFID Technology

The traditional manual attendance check-in or manual attendance check-in is widely used in colleges and universities. This method occupies a lot of time for teachers and is inefficient. RFID technology is used to collect student data, C/S architecture is used, and c# programming language is used to develop a card reader attendance management system. The student information is stored into the card reader database so that teachers can easily grasp the students' class situation. The system can greatly reduce the time spent on attendance, reduce the burden of teachers, and effectively improve the attendance rate of students. Before testing the college classroom attendance management system based on RFID technology, we need to understand the influence relationship between the number of readers and positioning performance. The simulation results are shown in Figure 3. As can be seen from the CDF distribution curve in the figure, when the number of readers is three, half of the probability of positioning error is not higher than 3.1 m; when the number of readers increases to four, half of the probability of positioning error is not higher than 2.35 m, and 80% of the probability is not higher than 3.2 m; when the number of readers increases to five, half of the probability of positioning error is no more than 2.2 m, and 80% of the probability is no more than 2.8 m.

Figure 4 shows the relationship between the number of readers and positioning accuracy in the Friis loss model. It can be seen from the data in the figure that when the number of readers is three, the probability of positioning error not exceeding 1.13 m is 50%, and the probability of not exceeding 1.2 m is 80%; after adding a reader, the probability of positioning error not higher than 0.89 m is 50%, and the probability of not higher than 0.94 m is 80%; when increasing to five readers, the probability of positioning error not higher than 0.84 m is half, and the probability of lower than 0.91 m is 80%.

To sum up, when the number of readers increases from three to four, the error decreases greatly, and the accuracy of system positioning is significantly improved. When it is increased from four to five, the decline of system error decreases, and the impact on accuracy is very small. Therefore, the increase of the number of readers will improve the positioning accuracy of the system, and the accuracy will increase with the increase of the number of readers. However, when the number of readers increases to a certain number, its further increase has little impact on the positioning accuracy of the system. Considering the actual situation, the number of readers is four, which is relatively appropriate.

As shown in Figure 5, the research results of user waiting time are queried by the university classroom attendance management system based on RFID technology. It can be seen from the data in the figure that 76% of users are satisfied that the time required for access query is 6 s; when the access query time increased to 11 s, the proportion of satisfied users decreased to 63%; when the access query time increased to 23 s, 41% of users were satisfied; only 5% of users said they could accept 36 s of query time. During the simulation experiment, the amount of database information of the system is relatively small and the number of users participating in the simulation test is limited. Therefore, the average query time is maintained at 5 s, which can basically meet the needs of all users. However, in a practical application, the number of users and database information will continue to increase, which will also increase the burden on the system operation. In case of slow operation, it is necessary to further optimize the system.

As shown in Figure 6, it is the relationship between the university classroom attendance management system based on RFID technology, response time, and server request. It can be seen from the figure that the increase in the number of login users will prolong the system response time. When the number of users increases to 100, the system response time is 30 times that of 20 users. The number of requests that the server can handle per unit time decreases with the increase of the number of users. When the number increases to 100, the number of requests processed by the server decreases by 14 compared with the initial number.

### 4.2. Test and Results of College Classroom Attendance Management System Based on Face Recognition Technology

The classroom attendance test results of college classroom attendance management system based on face recognition technology are shown in Figures 7 and 8; 1 in the figure indicates that the recognition of the student in the classroom is successful, and 0 indicates that the recognition is unsuccessful. It can be seen that the university classroom attendance management system based on face recognition technology can realize independent classroom attendance and identify the access of students in the classroom, such as leaving early, absenteeism, and substitute classes. Because the face recognition technology will be affected by the lighting conditions of the surrounding environment, students' sitting posture, expression, and other factors, although some students attend class on time, the system still shows that the recognition fails. On the whole, the test results of college classroom attendance management system based on face recognition technology are basically consistent with the sample results and can meet the expected requirements.

To sum up, both the university classroom attendance management system based on face recognition technology and the university classroom attendance management system based on RFID technology can basically meet the needs of classroom attendance with high accuracy. However, due to the limitations of technology and environment, both of them have some disadvantages. The college classroom attendance management system based on RFID technology cannot meet the needs of college students of different majors to log in to the system at the same time, and the running time will slow down with the increase of the number. The university classroom attendance management system based on face recognition technology has certain requirements for the environment of classroom attendance. Therefore, both of them need to be further optimized and improved.

## 5. Conclusion

This study presents the research of college intelligent classroom attendance management system based on the framework of Internet of things. Under the framework of Internet of things, this study constructs a classroom attendance management system based on RFID technology and face recognition technology. The experimental results show that the intelligent classroom attendance management system based on RFID technology can accurately identify students' absence and substitution. It has the advantages of fast response speed and low cost. The intelligent classroom attendance management system based on face recognition technology can accurately record and identify the situation of students entering and leaving the classroom and identify the situation of being late and leaving early, absenteeism, and substitute classes. The experimental results are basically consistent with the sample results, and the error rate is low. This study provides technical support for the development of Internet of things technology and the informatization reform of educational management in colleges and universities and makes the classroom attendance management in colleges and universities have a new development direction. The experimental results are basically consistent with the sample results. However, it is easily affected by ambient light, students' sitting posture, and expression and cannot be recognized. These two kinds of college classroom attendance management systems can meet the basic needs of colleges and universities, but there are still some technical limitations, which need to be further optimized and debugged.

## Figures and Tables

**Figure 1:** Overall block diagram of classroom attendance management system based on RFID technology.

**Figure 2:** Effect drawing of antiproxy brushing of college classroom attendance management system based on RFID technology.

**Figure 3:** The influence of the number of readers in the system on the positioning accuracy.

**Figure 4:** Effect of the number of readers in Friis loss model on positioning accuracy.

**Figure 5:** University classroom attendance management system based on RFID technology queries the research results of user waiting time.

**Figure 6:** RFID-based campus attendance management system's user number and response time relationship and server request relationship diagram.

**Figure 7:** Test results of college classroom attendance management system based on face recognition technology.

**Figure 8:** Comparison of attendance score and sample score in system experiment.

## Data Availability

The data used to support the findings of this study are available from the corresponding author upon request.
